The article "Severe congenital nemaline myopathy with primary pulmonary lymphangiectasia: unusual clinical presentation and review of the literature" was published in 2015. Journal: Diagn Pathol.

# Severe congenital nemaline myopathy with primary pulmonary lymphangiectasia: unusual clinical presentation and review of the literature

**DOI:** 10.1186/s13000-015-0270-8

**Published:** 2015-04-16

**Authors:** Jariya Waisayarat, Chinnawut Suriyonplengsaeng, Chaiyos Khongkhatithum, Mana Rochanawutanon

**Affiliations:** Department of Pathology, Faculty of Medicine Ramathibodi Hospital, Mahidol University, Bangkok, 10400 Thailand; Department of Pedriatrics, Faculty of Medicine Ramathibodi Hospital, Mahidol University, Bangkok, 10400 Thailand; Department of Anatomy, Faculty of Science, Mahidol University, Bangkok, 10400 Thailand

**Keywords:** Severe congenital nemaline myopathy, Congenital myopathy, *ACTA1*, Chylothorax, Primary pulmonary lymphangiectasia

## Abstract

**Introduction:**

Nemaline myopathy is a rare genetic muscle disorder defined by the presence of nemaline rods in the muscle fibre sarcoplasm. Congenital nemaline myopathy is the most serious form of the disease’s spectrum.

**Case presentation:**

The affected newborn has no spontaneous movement, fractures at birth and respiratory insufficiency. The present case was a Thai male, floppy at birth with fractures of both humeri and femurs and ventilator-dependent respiration. The patient developed bilateral chylothorax two weeks later and died at the age of 6 weeks. Whole-body postmortem examination with informed consent and genetic analysis of *ACTA1* mutation were performed. A skeletal muscle biopsy examined by light and transmission electron microscopy showed the features of nemaline myopathy. *ACTA 1* heterozygous missense mutation (c.1127G > C) was identified. Histological examination of both lungs revealed primary pulmonary lymphangiectasia.

**Conclusion:**

To the best of our knowledge, congenital nemaline myopathy with primary pulmonary lymphangiectasia causing bilateral chylothrax has never been previously reported. Considering chylothorax as a poor prognostic index and an unusual clinical presentation of severe congenital NM are proposed.

**Virtual Slides:**

The virtual slide(s) for this article can be found here: http://www.diagnosticpathology.diagnomx.eu/vs/9710506431489501.

## Background

The hallmark of all nemaline myopathies (NM), regardless of the genetic defect, is the presence of intrasarcoplasmic rod-like structures called nemaline bodies/rods which are stained red on the modified Gömöri trichrome preparation. This disorder was first recognized in 1963 by Shy and colleagues [1]. They proposed the term “nemaline myopathy” derived from the Greek word “nema” meaning thread. At the present time, NM is a well-recognized myopathy involving multiple genetic defects and encompassing a broad clinical spectrum varying from mild to severe muscle weakness. Affected patients are classified into six types based on the age at onset and the severity of motor and respiratory involvement according to the classification of Wallgren-Pettersson and colleagues [2,3]. Congenital nemaline myopathy is the most serious form of the disease’s spectrum. The affected newborn has no spontaneous movement, fractures at birth and respiratory insufficiency. Mutations in eight genes have now been identified in NM; *ACTA1, NEB, TPM2, TPM3, TNNT1, CFL2, KBTBD13* and *KLHL40* [4,5]. NM is listed as a “rare disease” by the Office of Rare Diseases of the National Institutes of Health. We present the postmortem examination of a case of congenital NM with the additional finding of bilateral chylothorax. Only two cases of severe congenital NM with chylothorax have been documented in the literature [6,7]. However, no cause of chylothorax was identified in both cases described in the literature. We discuss the possible mechanism of chylothorax in NM. Chylothorax is also a rare condition defined as the accumulation of chyle in the pleural space. Aetiologies of chylothorax can be mainly classified as traumatic or non traumatic [8]. Non traumatic causes are further subclassified as malignancy, diseases, congenital malformation or idiopathic. Moreover, congenital disorders and trauma due to intrathoracic surgery are responsible for the pathogenesis of neonatal chylothorax in most cases [9].

The article "Severe congenital nemaline myopathy with primary pulmonary lymphangiectasia: unusual clinical presentation and review of the literature" was published in 2015. Journal: Diagn Pathol.

## Case presentation

A male infant with generalized symmetrical hypotonia was born to non-consanguineous parents. The mother was a primigravida 22-year-old and the father was a healthy 28-year-old. Five older sisters and three older brothers of the maternal grandfather had died within the first year of life ranging from stillbirth to 7 months old without clarified cause of death. A cesarean section was carried out in the 37^th^ week of gestation because of breech presentation. Closed fractures of both humeri and femurs had occurred during delivery. Plaster casts were applied. The baby had absent spontaneous movement and difficult breathing. Apgar scores of 4 and 6 were documented at the 1^st^ and 5^th^ minutes, respectively. Eye movements were unimpaired. Intubation and ventilatory support were required. Weight, crown-heel-length and head circumference were within normal limits (2,750 g, 47 cm and 37 cm, respectively). Neurological deficits were observed; absent primitive reflexes (Moro, Babinski and grasping reflexes), loose anal sphincter tone and areflexia of all four limbs. Two weeks after birth, the patient developed bilateral pleural effusions (Figure 1) subsequently diagnosed as bilateral chylothorax due to the high triglyceride level (4,773 mg/dl) of the pleural fluid. No clinical evidence of heart failure was documented. Serum creatine kinase was normal (16 and 25 U/L). Spinal muscular atrophy was excluded by analysis of the *SMN* gene in which no mutations were found. Muscle biopsy from the right quadriceps femoris was performed at the age of 1 month. Despite the symptomatic treatment with ventilator support, intercostal drainage and parenteral nutrition, the patient still suffered from respiratory insufficiency and finally died at the age of 6 weeks. Informed consent for postmortem examination was formally obtained.

The article "Severe congenital nemaline myopathy with primary pulmonary lymphangiectasia: unusual clinical presentation and review of the literature" was published in 2015. Journal: Diagn Pathol.

**Figure 1:** Chest radiograph demonstrated bilateral pleural effusion at 2 weeks of age. Closed fractures of both humeri were noted.

### Postmortem examination

A high-arched palate and micrognathia were observed. Plaster casts of all fracture sites were noted. Generalized mild pitting oedema was present. Internal examination of the thoracic cavity revealed minimal milky fluid in both pleural cavities and severe pleural adhesions. The lung weight (60 g in total) and anatomy were normal. The thoracic duct rupture was not apparent. The cut surfaces of both lungs showed many dilated spaces measuring up to 0.2 cm in diameter. No structural cardiac anomaly was observed. Both testes were identified at the internal openings of the inguinal canals. Brain examination showed a normal external configuration with mild non-obstructive hydrocephalus revealed on slicing. Muscle samples from the biceps brachii, intercostal muscles, diaphragm and quadriceps femoris were obtained.

### Microscopic examination

All muscle tissue obtained before and after death were preserved using a snap freezing technique. Frozen sections (10 microns) were cut and stained using a panel of tinctorial and enzyme histochemical methods according to standard protocols; haematoxylin and eosin (H&E), modified Gömöri trichrome (mGt), nicotinamide adenine dinucleotide - tetrazolium reductase (NADH-TR), cytochrome oxidase (COX), succinate dehydrogenase (SDH), COX/SDH, periodic acid-Schiff (PAS), PAS with diastase (PASD), oil red O, myophosphorylase, alkaline phosphatase, adenylate deaminase and ATPase at pH 4.3, 4.6 and 9.4.

Routine histology of the muscle demonstrated well populated fascicles and marked variation in muscle fibre size (4-40 micron). There were mild increase in internal nuclei (6% of fibres), scattered atrophic and regenerating fibres, and moderate increase in endomysial and perimysial connective tissue. Split, whorled, necrotic and ragged red fibres were absent. Numerous nemaline rods were highlighted with mGt staining in almost type I fibres (Figure 2A). Transmission electron microscopy demonstrated copious sarcoplasmic electron dense nemaline rods (Figure 2B). Rods appeared either as extensions of sarcomeric Z-lines, in random array without obvious attachment to Z-lines, or in large clusters localized at the sarcolemma or intermyofibrillar spaces. The diagnosis of nemaline myopathy was established considering the clinical presentation and muscle pathology. Routine histology of the sampled tissue from each organ was performed. Microscopic examination of both lungs showed mature alveoli compatible with the alveolar stage of lung development. Diffuse dilatation of existing lymphatic vessels, without an increase in their number or complexity, were bilaterally evident in the subpleural connective tissue, interlobular septa and peribronchovascular areas (Figure 2C, D). The appearance was compatible with pulmonary lymphangiectasia rather than lymphangiomatosis. Positive immunoreactivity for CD31 and CD34 (low level) of the endothelial cells lining dilated lymphatic vessels was demonstrated. The hyaline membrane, a feature of diffuse alveolar damage, was absent. The CD31-and-CD34-immunoreactive endothelium of the dilated lymphatic vessels was also identified in the sections of pancreas. A choroid plexus papilloma 1 cm in diameter with features of a WHO grade I lesion was present in the left lateral ventricle giving rise to the documented communicating hydrocephalus.

The article "Severe congenital nemaline myopathy with primary pulmonary lymphangiectasia: unusual clinical presentation and review of the literature" was published in 2015. Journal: Diagn Pathol.

**Figure 2:** Summary of investigation. (**A**) The quadriceps femoris biopsy showed multiple red nemaline rods in sarcoplasm. mGt, X1000. (**B**) Electron micrograph revealed many nemaline rods (arrow) of uneven size. X30000. (**C**) Dilated lymphatic vessels (star) were noted in the pleura and interlobular septum. H&E, X100. (**D**) Low power demonstrated markedly-dilated lymphatic vessels (star) in peribronchovascular areas. Some were more than 5 times of the adjacent alveolar diameter. H&E, X40. (**E**) Normal sequence of the *ACTA 1* gene (control). (**F**) A heterozygous substitution of G to C at nucleotide position 1127 (c.1127G > C) in exon 7 of *ACTA1* gene was evident.

### Genetic analysis

*ACTA1* gene analysis was performed on DNA derived from blood. Mutation analysis in 6 coding exons (exon 2-7) of *ACTA1* gene was performed by PCR amplification, followed by direct DNA sequencing. A heterozygous substitution of G to C at nucleotide position 1127 (c.1127G > C) in exon 7 of *ACTA1* was identified, resulting in a Cys to Ser substitution at codon 376 (Cys376Ser) (Figure 2E,F). No *ACTA1* mutation was evident in blood samples from either parent.

## Discussion

The *ACTA1* gene locating on chromosome 1 (1q42.13) normally encodes skeletal muscle α-actin protein, which is an essential component of sarcomeres in skeletal muscle fibres. Actin proteins are not only important for cell movement and muscle contraction, but also help maintaining the cytoskeleton determining cell shape and organizing cellular contents. Mutation of *ACTA1* results in various types of congenital myopathy. *ACTA1* heterozygous missense mutation combined with the microscopic finding of nemaline rods in the sarcoplasm warrants the diagnosis of NM in the present case. This genetic defect represents a dominant mutation arising de novo as neither parent carried the mutation. This pattern of inheritance is commonly identified in NM cases caused by the mutation in *ACTA1* [4,10,11].

The article "Severe congenital nemaline myopathy with primary pulmonary lymphangiectasia: unusual clinical presentation and review of the literature" was published in 2015. Journal: Diagn Pathol.

Due to the absence of spontaneous neonatal movement, respiratory insufficiency and fractures of both humeri and femurs at birth, NM in this patient was categorized as the severe congenital type [2,3]. The disease caused additional neurological deficits (absent primitive reflexes, loose anal sphincter tone and areflexia of all extremities). The affected diaphragm, confirmed by the presence of numerous nemaline rods, resulted in the ventilator-dependency from birth. This respiratory insufficiency was well correlated with the study data of Ryan MM and colleagues [3] in that all 23 reviewed cases with severe congenital NM had significant respiratory problems and twelve were ventilator-dependent.

Pulmonary pathology consisted of diffuse bilateral pulmonary lymphangiectasia. Absent clinical signs and symptoms of heart failure and passive congestion of liver and spleen supported the diagnosis of primary or congenital pulmonary lymphangiectasia (PPL). PPL is a rare congenital disease of unknown cause characterized by abnormal pulmonary lymphatic dilatation in the absence of secondary lymphatic obstruction [12]. Bilateral chylothorax had been clinically observed in the present case. Chylothorax is defined as the accumulation of lymphatic fluid in the pleural space. In neonatal chylothorax both congenital and traumatic (especially after thoracic surgery) forms have been recognized. Congenital chylothorax in some cases is associated with Turner syndrome, Noonan syndrome, Down syndrome, congenital lymphangiectasia or hydrops fetalis [9]. Despite no obvious evidence of microscopic pleural rupture in this case, the most likely cause of the bilateral chylothorax was PPL. The association between PPL and congenital chylothorax had been well documented [13,14]. Neonatal onset PPL without additional anomalies is now compatible with life and has a good prognosis in the ventilator era of neonatal intensive care [12]. In this case PPL with chylothorax may have been aggravated by the hypotonic diaphragm due to NM. Prolonged intubation since birth causing compression to the thoracic duct leading to increased hydrostatic pressure in the thoracic duct and subsequent chylous leakage is another possible additional cause of chylothorax in the present case.

The article "Severe congenital nemaline myopathy with primary pulmonary lymphangiectasia: unusual clinical presentation and review of the literature" was published in 2015. Journal: Diagn Pathol.

Our case represents the third example of severe congenital NM with chylothorax to be documented in the literature [6,7], however, the etiology of chylothorax in those two cases has yet to be established. To the best of our knowledge, severe congenital NM with PPL causing bilateral chylothrax has never been previously reported. Two further cases of congenital myopathy (myotubular myopathy, congenital myotonic dystrophy type 1) with chylothorax of unknown cause have also been reported [15,16]. The reported cases are summarized in Table 1. All 3 reported cases of NM with chylothorax were male with severe congenital presentation of myopathy and de novo dominant mutation in *ACTA1*. Among these three cases of NM with chylothorax, none survived more than 9 weeks indicating a poor prognosis in this group and suggesting that this represents a poor prognostic sign. Moreover, recognition that chylothorax can be an unusual clinical manifestation of severe congenital NM, or other myopathies, indicates that myopathy should be included in the differential diagnosis of chylothorax in the neonate.

**Table 1:** **Clinical data of case reports of congenital myopathy with chylothorax**

**Study**	**Authors’ study**	**Garcia-Angarita, et al. (2009) [** 7 **]**	**Schröder, et al. (2004) [** 6 **]**	**Smets (2008) [** 15 **]**	**Son, et al. (2012) [** 16 **]**
**Age at presentation**	At birth (GA 37 week)	At birth (GA 39 week)	At birth	At birth	At birth, (GA 30 week, non-identical twin A)
**Sex**	Male	Male	Male	Male	Male
**Race**	Thai	German	Turkish	Turkish	Korean
**Diagnosis**	Nemaline myopathy, severe congenital	Nemaline myopathy, severe congenital	Nemaline myopathy (intranuclear rod variant), severe congenital	Myotubular myopathy, severe congenital	Congenital myotonic dystrophy type 1
**Gene muatation**	*ACTA1* gene (c.1127G > C, exon 7), heterozygous	*ACTA1* gene (c.222G > T & c.223C > T, exon 3), heterozygous	*ACTA1* gene (Asp154Asn, exon 4), heterozygous	*MTM1* gene (c.1261-10A > G)	*DMPK* gene (more than 750 CTG repeats)
**Inheritance**	De novo	De novo	De novo	X-linked recessive	Autosomal dominant (affected mother)
**Chylothorax**	Bilateral	Bilateral	Present	Bilateral	Bilateral
**Triglyceride level in pleural effusion (mg/dl)**	4773	NA	NA	746	495
**Cause of chylothorax**	Primary pulmonary lymphangiectasia	Not defined	Not defined	Not defined	Not defined
**Serum creatine kinase (U/L)**	16-25, Low, (normal 30-200 U/L)	Normal	NA	NA	281
**Signs and symptoms**	Absent spontaneous neonatal movement, respiratory difficulty, fractures of both humeri and femurs, high arch palate	Absent spontaneous neonatal movement, respiratory difficulty, fractures of both humeri and femurs	Generalized hypotonia, respiratory difficulty, right pulmonary hypoplasia	Generalized hypotonia, respiratory difficulty	Generalized hypotonia, respiratory difficulty, triangular face, inverted v-shaped upper lip
**Age at death, Cause of death**	6 weeks, respiratory failure	8 weeks, respiratory failure	9 weeks, respiratory failure	16 weeks, NA	14 weeks, respiratory failure and pneumonia

GA, gestational age; NA, not available.

The article "Severe congenital nemaline myopathy with primary pulmonary lymphangiectasia: unusual clinical presentation and review of the literature" was published in 2015. Journal: Diagn Pathol.

## Conclusion

We report a case of congenital nemaline myopathy presenting with classical features of the disease (fractures, respiratory insufficiency and absence of spontaneous movement at birth) combined with unusual presentation (bilateral chylothorax due to primary pulmonary lymphangiectasia). The presence of nemaline rods in the skeletal muscle biopsy examined by light and electron microscopy, and *ACTA1* mutation analysis (c.1127G > C) confirmed this muscular disorder. Lung histological examination revealed diffuse dilatation of existing lymphatic vessels. Together with the absence of secondary causes, this lung pathology was diagnosed as primary pulmonary lymphangiectasia. Recognition that chylothorax can be an unusual clinical manifestation of severe congenital NM, or other myopathies, indicates that myopathy should be included in the differential diagnosis of chylothorax in the neonate.

## Consent

Written informed consent was obtained from the patient’s parent for publication of this case report and any accompanying images. A copy of the written consent is available for review by the Editor-in-Chief of this journal.

## Abbreviations

*ACTA1*: Alpha-skeletal actin gene
COX: Cytochrome oxidase
H&E: Haematoxylin and eosin
mGt: Modified Gömöri trichrome
NADH-TR: Nicotinamide adenine dinucleotide-tetrazolium reductase
NM: Nemaline myopathy
PAS: Periodic acid-Schiff
PASD: PAS with diastase
PPL: Primary or congenital pulmonary lymphangiectasia
SDH: Succinate dehydrogenase
